The article "Effect of Different Hemodialysis Methods on Microbiota in Uremic Patients" was retracted in 2024. Reasons: signs of a paper mill; suspected computer-generated content; unreliable results or conclusions; concerns about the data.

# Effect of Different Hemodialysis Methods on Microbiota in Uremic Patients

**DOI:** 10.1155/2020/6739762

**Published:** 2020-06-19

**Authors:** Haidong He, Yan Xie

**Affiliations:** ^1^Department of Geriatrics, First Affiliated Hospital of Soochow University, No. 899, Pinghai Road, 215006 Suzhou, China; ^2^Minhang Hospital, Fudan University, Shanghai, China

## Abstract

**Background:**

To investigate the effect of hemodialysis on microbiota in uremic patients.

**Objective:**

To investigate the effect of hemodialysis on microbiota in uremic patients.

**Methods:**

This study included 85 adult patients who have received hemodialysis since August 2014, and the treatment plan has not changed for more than 12 months. These patients were divided into hemodialysis group (group A), hemodialysis+hemodialysis filtration group (group B), and hemodialysis+hemodialysis filtration+blood perfusion group (group C). Twenty-four adult ESRD patients (CK group) were enrolled. Serum biochemical indexes were measured, glomerular filtration rate (EGFR) was estimated, dialysis adequacy (kt/V) was calculated, and fresh feces were collected. At the same time, the feces of 30 health workers were selected as the control. 16S rRNA sequence was used to determine the intestinal flora of all fecal specimens. First of all, we analyzed the difference of the whole flora distribution between dialysis and nondialysis ESRD patients; then, we selected the most representative content of bifidobacteria, *Lactobacillus acidophilus*, *Escherichia coli*, and *Enterococcus faecalis* to analyze the influence of different blood purification methods on the intestinal flora.

**Results:**

(1) The level of C-reactive protein (CRP) in dialysis patients was lower than that in nondialysis ESRD patients, and CRP in group C was lower than that in groups A and B. There was no significant difference in kt/V between group A, group B, and group C. There was no significant difference in EGFR between the four groups. (2) The species diversity of ESRD patients without dialysis (CK group) was significantly lower than that of ESRD patients with dialysis; there was no significant difference between group A and group B; the species diversity of group C was significantly higher than that of group A and group B. (3) Compared with the control group, the levels of bifidobacteria and *Lactobacillus acidophilus* in ESRD patients were significantly lower, while the levels of *Escherichia coli* and *Enterococcus faecalis* were significantly higher. (4) The levels of bifidobacteria and *Lactobacillus acidophilus* in hemodialysis patients were significantly higher than those in nonblood purification treatment group, and the levels of *Escherichia coli* and *Enterococcus faecalis* were significantly lower than those in nonblood purification treatment group. (5) The level of *Lactobacillus acidophilus* in group C was significantly higher than that in groups A and B, and the level of *Escherichia coli* was significantly lower than that in groups A and B.

The article "Effect of Different Hemodialysis Methods on Microbiota in Uremic Patients" was retracted in 2024. Reasons: signs of a paper mill; suspected computer-generated content; unreliable results or conclusions; concerns about the data.

**Conclusion:**

ESRD patients have microbiota disorder. Hemodialysis can improve microbiota disorder in uremic patients. Compared with ordinary hemodialysis, combined hemoperfusion dialysis can further improve microbiota disorder.

## 1. Introduction

Chronic kidney disease (CKD) is a common chronic disease in the world, affecting millions of people around the world [1]. Part of chronic nephropathy can gradually progress to end-stage renal disease (ESRD), that is, uremia. At this stage, patients may need to rely on renal replacement therapy, such as hemodialysis (hd), hemodialysis filtration (HDF), hemoperfusion (HP), peritoneal dialysis (PD), and kidney transplantation.

For ESRD patients, the most common cause of death is cardiovascular disease (CVD). The increased risk of cardiovascular death in patients with chronic kidney disease is not only attributed to traditional risk factors, such as hypertension, diabetes, and dyslipidemia, but also to nontraditional risk factors [2]. Among the nontraditional risk factors, chronic inflammation has attracted more and more attention and is recently considered as the main catalyst of CVD in chronic kidney disease [3]. There is a close relationship between intestinal environment and kidney disease in patients with CKD. And there are negative effects of uremic toxins on the structure and function of intestinal barrier, especially on the structure/function of closely linked proteins [4]. In the absence of clinical infection, inflammatory molecules and toxins from the gut to the blood (translocation of intestinal flora) may trigger and/or enhance the inflammatory state of CKD/ESRD [5]. Therefore, this study will focus on the patients with uremia to understand the changes of intestinal flora and the effect of hemodialysis on intestinal flora.

## 2. Materials and Methods

### 2.1. Subjects

The study included 85 adult patients who had received hemodialysis since August 2014, and the treatment plan had not changed for more than 12 months. These patients were divided into several groups: (1) simple hemodialysis group (group A) (*n* = 30), hemodialysis+hemodialysis filtration group (group B) (*n* = 29), and hemodialysis+hemodialysis filtration+blood perfusion group (group C) (*n* = 26). In addition, another 24 adult ESRD patients (CK group) who did not receive any renal replacement therapy were selected. At the same time, the feces of 30 health medical staff were taken as health control. Exclusion criteria: patients who had received other renal replacement therapy before the study, such as peritoneal dialysis and kidney transplantation, were excluded. Other exclusion criteria include clinical infection (respiratory tract, digestive tract, urogenital system, etc.), liver disease, autoimmune disease, malignant tumor, congestive heart failure, diarrhea, or constipation. Patients who received antibiotics or probiotics/prebiotics within the first three months of the study were also excluded. Try to keep the normal eating habits one week before sampling; do not change the diet greatly; women in physiological period cannot sample; collect morning stool; and avoid urine pollution.

The article "Effect of Different Hemodialysis Methods on Microbiota in Uremic Patients" was retracted in 2024. Reasons: signs of a paper mill; suspected computer-generated content; unreliable results or conclusions; concerns about the data.

Hemodialysis program: group A: receiving HD treatment, 3 times a week; group B: HD twice a week, HDF once a week, 4H each time; group C: HD+Hp once a week, HD+Hp once a week (1.5-2 hours HP+HD treatment, 2-2.5 hours HD treatment), HD once, HDF once a week. The hemoperfusion device is the ha130 resin perfusion device produced by Zhuhai Jianfan Biotechnology Co., Ltd. The vascular access is arteriovenous fistula or semipermanent hemodialysis catheter, all of which are anticoagulant with low molecular weight heparin, dialysis water with reverse osmosis, and bicarbonate dialysate. The dialysate flow rate is 500 mL/min, and the dialysate flow rate is maintained at 200-250 mL/min. According to the individual situation, erythropoietin, iron, active vitamin D, phosphorus binding agent, and antihypertensive drugs are routinely used.

### 2.2. Data Collection

All the participants collected venous blood samples in the morning when they were fasting to detect the levels of hemoglobin (Hb), serum albumin (Alb), blood phosphorus (P), blood calcium (Ca), whole parathyroid hormone (iPTH), high-sensitivity C-reactive protein (hs-CRP), serum creatinine (Scr), and blood urea nitrogen (BUN); group A patients detected Scr and BUN after hemodialysis. The indexes of dry weight, height, ultrafiltration volume, and dialysis time were recorded. The dialysis adequacy (kt/V) was calculated by Daugirdas formula: kt/*v* = −ln (*r* − 0.008 × *T*) + (4 − 3.5 × *R*) × UF/*W*, (ln: natural logarithm; t: time of each dialysis; R: the ratio of bun concentration after dialysis and before dialysis; UF: ultrafiltration volume; W: the weight of patients after dialysis).

Using MDRD simplified formula to evaluate glomerular filtration rate (eGFR): 186 × [Scr (mg/dL)]^−1.54^ × [age (year)]^−0.203^ × (0.742female)[mL/(min•1.73 m^2^)].

### 2.3. 16S rRNA Sequencing

The first fresh stool in the morning was collected and stored at -80°C. Stool DNA was extracted using a QIAamp Fast DNA Stool Mini kit (Qiagen, Germantown, MD, USA) according to the manufacturer's instruction. A total of 4 well-known bacteria were chosen in this study, *Bifidobacterium*, *Lactobacillus acidophilus*, *Escherichia coli*, and *Enterococcus faecalis*. RNA was converted into cDNA using a Prime-ScriptTM one step qRT-PCR kit (TAKARA, Dalian, China). PCR reactions were performed with using SYBR GREEN mastermix (Solarbio, Beijing, China) on an ABI7500System (Applied Biosystems, Foster City, CA, USA) with the following composition and cycling profile: predenaturation at 95°C for 2 minutes, then denaturation at 95°C for 15 seconds; annealing for 20 seconds 58°C for *Bifidobacterium*, 58°C for *Lactobacillus acidophilus*, 60°C for *Escherichia coli*, and 61°C for *Enterococcus faecalis*; 68°C for 30 seconds, and 15 seconds of 85°C for *Bifidobacterium*, 83.5°C for *Lactobacillus acidophilus*, 85.5°C for *Escherichia coli*, and 82.5°C for *Enterococcus faecalis*. A total 40 cycles were conducted. The 16S rDNA primers are designed and synthesized by the Beijing Genomics Institute Inc. Sequences were as follows: *Bifidobacterium* F 5′-TCGCGTC(C/T)GGTGTGAAAG-3′, R 5′-CCACATCCAGC(A/G)TCCAC-3′; *Lactobacillus acidophilus* F 5′-AGCAGTAGGGAATCTTCCA-3′, R 5′-CACCGCTACACATGGAG-3′; *Escherichia coli* F 5′-CCCTTATTGTTAGTTGCCATCATT-3′, R 5′-ACTCGTIGTACTTCCCATTGT-3′; *Enterococcus faecalis* F 5′-GTTAATACCTTTGCTCATTGA-3′, R 5′-ACCAGGGTATCTTAATCCTGTT-3′. Bacterial quantity was expressed as log10 bacteria per gram of stool.

The article "Effect of Different Hemodialysis Methods on Microbiota in Uremic Patients" was retracted in 2024. Reasons: signs of a paper mill; suspected computer-generated content; unreliable results or conclusions; concerns about the data.

### 2.4. Statistical Analysis

The measurement data was present as mean ± SD (standard deviation). Comparisons were conducted using one-way analysis of variance (ANOVA) followed by Tukey post hoc test. It was considered to be statistically significant when the *P* value was less than 0.05. The *P* value had been adjusted by FDR (false discovery rate). Fold change (>2 or <0.5) had been calculated to determine if the difference has changed. All calculations are made using SPSS 18.0 (SPSS Inc.; Chicago, IL, USA) [6].

## 3. Results

### 3.1. Basic Characteristics

As shown in Table 1, a total of 109 patients were included in this study with 85 cases having received hemodialysis with a mean age of 56.8 ± 15.5 and male : female ratio of 44 : 41, while 24 cases in the nonhemodialysis group had a mean age of 57.2 ± 15.1 and male : female ratio of 14 : 11. Among all 109 patients, the cause for renal failure was chronic glomerulonephritis for 58 cases (53%), diabetic nephropathy for 23 cases (21%), hypertensive nephropathy for 9 cases (8%), medicinal nephropathy for 9 cases (8%), polycystic kidney for 6 cases (6%), and other types for 4 cases (4%). No significant difference was found in age, gender, and causes for renal failure in the patient groups.

The article "Effect of Different Hemodialysis Methods on Microbiota in Uremic Patients" was retracted in 2024. Reasons: signs of a paper mill; suspected computer-generated content; unreliable results or conclusions; concerns about the data.

There were no significant differences in hemoglobin (HB), albumin (ALB), glomerular filtration (EGFR), blood phosphorus (P), blood calcium (CA), whole parathyroid hormone (iPTH), and dialysis adequacy (kt/V) between the three groups, and there were significant differences between the three groups. There was no significant difference in CRP between group A (hd) and group B (HD+HDF). CRP in group C (HD+HDF+Hp) was significantly lower than that in group A and group B, and CRP in group A, group B, and group C were significantly lower than that in the nondialysis group.

### 3.2. 16S rDNA Sequencing Results

#### 3.2.1. Rarefaction Curve

The results showed that the species diversity of ESRD patients without dialysis (CK group) was significantly lower than that of ESRD patients with dialysis; there was no significant difference between group A and group B; the species diversity of C group was significantly higher than that of groups A and B (Figure 1).

#### 3.2.2. Stars diagram

As shown in Figure 2, the bacterial colony structure of ESRD patients receiving dialysis treatment was significantly more than that of ESRD patients without dialysis treatment.

#### 3.2.3. Error Bar

#### 3.2.4. Anosim Analysis

As shown in Figure 3, bifidobacteria and *Lactobacillus acidophilus* in CK group were significantly lower than those in ESRD group, while *Escherichia coli* and *Enterococcus faecalis* were significantly higher than those in other groups. *Lactobacillus acidophilus* in group C was significantly higher than that in groups A and B, while *Escherichia coli* was significantly lower than that in groups A and B.

It can be seen from Figure 4 that there are significant differences in colony distribution between the CK group and the dialysis group; there are also significant differences in colony distribution among the three groups of patients with different dialysis methods.

To further investigate the influence of uremia and treatment of hemodialysis on intestinal microflora, 4 well-known bacteria were chosen (as shown in Figure 3), *Bifidobacterium*, *Lactobacillus acidophilus*, *Escherichia coli*, and *Enterococcus faecalis*, and 16S rRNA sequence was quantitatively determined by RT-qPCR. At the same time, the results were compared with those of healthy people.

As shown in Figure 5, the levels of *Bifidobacterium* and *Lactobacillus acidophilus* were significantly lower in both of the patient groups compared with the healthy control, *P* < 0.05. However, the levels of *Escherichia coli* and *Enterococcus faecalis* were significantly higher in both of the patient groups compared with the healthy control, *P* < 0.05. Meanwhile, in all treatment groups, the levels of *Bifidobacterium* and *Lactobacillus acidophilus* were significantly higher, and levels of *Escherichia coli* and *Enterococcus faecalis* were significantly lower in hemodialysis patients compared with the nonhemodialysis treatment group, *P* < 0.05. The level of *Lactobacillus acidophilus* was significantly higher while *Escherichia coli* was significantly lower in the HD+HDF+HP group than HD and HD+HDF groups, *P* < 0.05. No other significant difference was observed between the two groups of HD and HD+HDF.

The article "Effect of Different Hemodialysis Methods on Microbiota in Uremic Patients" was retracted in 2024. Reasons: signs of a paper mill; suspected computer-generated content; unreliable results or conclusions; concerns about the data.

## 4. Discussion

C-reactive protein is mainly produced by the liver, which is part of the initial response of the immune system to inflammation. There are differences between dialysis and nondialysis patients, which can be used as auxiliary diagnostic indicators. The difference of intestinal microflora also exists between dialysis and nondialysis patients. Although there are similar studies on intestinal flora in many diseases, there are few studies on uremia. The molecular mechanism of intestinal microflora has not been understood, so this phenomenon is worthy of further study.

When CKD develops to ESRD stage, there will be multiple organ damage. CVD is the main cause of death. The risk factors of CVD in ESRD patients include not only hypertension, diabetes, and dyslipidemia in nonnephrotic patients but also nontraditional risk factors [2]. Especially in recent years, with the development of many researches, more and more attention has been paid to the microinflammation in CKD/ESRD patients. We know that intestinal flora is involved in the occurrence and progression of many diseases, including kidney diseases, especially in the CKD/ESRD period. The most direct consequence of intestinal disorder in CKD/ESRD period is bacterial translocation, endotoxin release into the blood [7], and intestinal catabolic products are absorbed by various toxin diseases, triggering and/or enhancing inflammatory response.

In CKD/ESRD, harmful bacteria such as *E. coli* [8, 9] will grow excessively, and beneficial bacteria such as lactobacilli will decrease [8]. Meanwhile, the number of bacteria containing urease will increase greatly, and their functions will increase significantly [10]. Therefore, the ability of gut to decompose toxins is significantly enhanced. In addition, the amount of urea discharged into intestinal cavity by CKD patients is increased, and the amount of ammonia and other harmful substances produced by microbial urease hydrolysis is significantly increased. These harmful substances not only damage the intestinal mucosal barrier [11, 12] but also are closely related to the occurrence of CVD [13, 14].

The article "Effect of Different Hemodialysis Methods on Microbiota in Uremic Patients" was retracted in 2024. Reasons: signs of a paper mill; suspected computer-generated content; unreliable results or conclusions; concerns about the data.

In our study, ESRD patients, whether receiving hemodialysis or not, had a disorder of intestinal flora. The sequencing results showed that the harmful bacteria such as Enterobacteriaceae grew excessively and the beneficial bacteria such as *Lactobacillus* decreased significantly, which were consistent with many literatures. The effect of different bacterial groups on renal function has been reported in many studies. For example, Ando et al. found the effect of oral *Bifidobacterium longum* enteric coated capsules on the progress of chronic renal failure [15]; Yoshifuji et al. reported in 2016 that *Lactobacillus entericus* can prevent the progress of renal damage by regulating the intestinal environment of rats [16]; Langenberg et al. also found that *E. coli* can have an impact on septic acute renal failure [17].

After recognizing the physiological function and pathological mechanism of intestinal flora, many researchers have explored various ways to reconstruct healthy intestinal flora, hoping to regulate intestinal flora, block lipopolysaccharide or reduce inflammation, or target to absorb enterotoxins fermented by microorganisms. There are common methods such as prebiotics, probiotics, and fecal bacteria transplantation and absorption of enterogenous uremic toxins. However, the application of these methods is limited by various factors, and the results are not satisfactory. In short, in terms of the current situation, there are no better clinical measures to improve the intestinal flora disorder and reduce the consequences of the flora disorder.

For ESRD patients with hemodialysis, the highest compliance is to receive hemodialysis treatment on time. Now, the progress of medical technology provides a variety of effective hemodialysis technology and equipment, so that ESRD patients' survival time and dialysis quality continue to improve. Compared with the conventional hemodialysis method, hemoperfusion (HP) is to introduce the blood into the absorption perfusion with solid adsorbent by means of cardiopulmonary bypass to absorb the toxins in a specific amount range, so as to achieve better blood purification effect. It has unique features in the removal of medium molecular substances [18, 19]. Hemodialysis combined with hemoperfusion is equivalent to combined artificial kidney (also known as combined hemodialysis), which not only enhances the elimination of toxins in vivo but also reduces the microinflammatory state in uremic patients. This study also confirmed that combined hemodialysis can reduce the inflammatory factors in ESRD patients. In this study, we investigated the effect of blood purification on intestinal flora in uremic patients. There were significant differences in colony distribution among patients with different dialysis methods. The level of *Lactobacillus acidophilus* in hemodialysis+hemodiafiltration+hemoperfusion group was significantly higher than that in hemodialysis group and hemodialysis+hemodiafiltration group, and the level of *Escherichia coli* was significantly lower than that in hemodialysis group and hemodialysis+hemodiafiltration group. We conclude that combined hemodialysis can provide more adequate dialysis effect, significantly reduce inflammatory factors, and possibly provide better bacterial abundance by improving the microinflammatory state in the body, which indicates that different hemodialysis methods have different effects on improving intestinal flora disorder. Therefore, we can improve the dialysis effect and promote more effective dialysis methods by means of hemodialysis, which may have a positive effect on improving intestinal flora disorder, so as to achieve the purpose of improving prognosis and reducing complications.

The article "Effect of Different Hemodialysis Methods on Microbiota in Uremic Patients" was retracted in 2024. Reasons: signs of a paper mill; suspected computer-generated content; unreliable results or conclusions; concerns about the data.

Several limitations should be noted in this study. First, clinical samples used in this study are limited. In the future study, our follow-up study on uremia will continue using more clinical samples. Second, we should further explore whether different hemodialysis methods affect the changes of other microbiome in patients with uremia. Third, we should perform several functional analyses to determine the effects of bifidobacteria, *Lactobacillus acidophilus*, *E. coli*, and *Enterococcus faecalis* on renal function. Further demonstrating these limitations could provide more information to understand the effect of hemodialysis on microbiota in uremic patients.

## 5. Conclusion

We investigated alterations of intestinal microflora in uremia patients with or without blood purification and found that the intestinal microflora might be influenced by uremia and may be affected by blood purification treatments. Further studies would be still needed to confirm our results. Our result of the study has explored uremia from different perspectives, providing help for treatment and diagnosis.

## Figures and Tables

**Figure 1:** Dilution curve. Species diversity of ESRD patients. The abscissa represents the number of sequences randomly selected from the sample, and the ordinate represents the theoretical number obtained from analysis and analysis after extraction. ^∗^*P* < 0.05 compared with the ESRD patients with dialysis, and #*P* < 0.05 compared with group A and group B.

**Figure 2:** Results of stars. Bacterial colony structure of ESRD patients. Group A, group B, group C and group CK are shown in from the first line down. The size of the sector represents the size of species richness, and the color of the sector represents different species.

The article "Effect of Different Hemodialysis Methods on Microbiota in Uremic Patients" was retracted in 2024. Reasons: signs of a paper mill; suspected computer-generated content; unreliable results or conclusions; concerns about the data.

**Figure 3:** Comparison histogram of flora. Each column (group) represents the relative abundance of a species, and the bacteria with differences between groups are marked in red font. The thin line at the top is error bar (1 SD). ^∗^*P* < 0.05 vs. group A, group B, and group C. #*P* < 0.05 vs. group A and group B.

**Figure 4:** Anosim analysis results. *Between* represents the difference between groups; others are within groups; the greater the distance is, the greater the difference is; and the thickness is the sample size.

**Figure 5:** Levels of *Bifidobacterium*, *Lactobacillus acidophilus*, *Escherichia coli*, and *Enterococcus faecalis*.Effect of different hemodialysis methods on intestinal flora. ^∗^*P* < 0.05.

**Table 1:** Basic characteristics.

Patients	Group A (HD) *n* = 30	Group B (HD+HDF) *n* = 29	Group C (HD+HDF+HP) *n* = 26	Group CK (nondialysis) *n* = 24
Age (years)	56.3 ± 13.6a	57.6 ± 12.1ac	55.4 ± 16.2acd	57.2 ± 15.1
Gender male : female	16 : 14a	15 : 14ac	13 : 13acd	12 : 12
Cause of renal failure *n* (%)				
Chronic glomerulonephritis	16 (53)a	15 (52)ac	15 (58)acd	12 (50)
Diabetic nephropathy	7 (23)a	7 (24)ac	5 (19)acd	4 (17)
Hypertensive nephropathy	3 (10)a	2 (7)ac	2 (8)acd	2 (8)
Medicinal nephropathy	2 (7)a	2 (7)ac	3 (12)acd	2 (8)
Polycystic kidney	2 (7)a	1 (3)ac	2 (8)acd	1 (4)
Other	1 (3)a	1 (3)ac	1 (4)acd	1 (4)
Duration for hemodialysis	5.1 ± 3.1	5.2 ± 2.6c	5.0 ± 3.3cd	
Hb (g/L)	101.4 ± 15.3b	101.2 ± 17.7bc	103.4 ± 16.1bcd	88.9 ± 13.6
Alb (g/L)	39.4 ± 7.4b	39.7 ± 9.5bc	40.9 ± 8.4bcd	32.3 ± 8.9
CRP (mg/L)	10.2 ± 0.9b	10.1 ± 1.2bc	7.1 ± 1.1bcef	27.2 ± 1.0
Ca (mmol/L)	2.41 ± 0.21a	2.50 ± 0.30ac	2.45 ± 0.18acd	2.47 ± 0.20
P (mmol/L)	1.75 ± 0.33a	1.71 ± 0.28ac	1.68 ± 0.13acd	1.74 ± 0.24
iPTH (pg/mL)	325.12 ± 22.4a	298.6 ± 17.8ac	302.6 ± 23.5acd	325.12 ± 30.8
eGFR (mL/min)	6.9 ± 3.0a	7.1 ± 2.8ac	7.4 ± 3.7acd	7.3 ± 2.4
KT/V	1.25 ± 0.1	1.28 ± 0.3c	1.28 ± 0.2cd	

Hb: hemoglobin; Alb: albumin; Scr: serum creatinine; BUN: blood urea nitrogen; eGFR: estimated glomerular filtration rate. ^a^*P* > 0.05 vs. group CK; ^b^*P* < 0.05 vs. group CK; ^c^*P* > 0.05 vs. group A; ^d^*P* > 0.05 vs. group B; ^e^*P* < 0.05 vs. group A; ^f^*P* < 0.05 vs. group B.

## Data Availability

The data used to support the findings of this study are available from the corresponding author upon request.
